The article "Clinical Diagnosis, Treatment, and Laboratory Detection of 50 Cases of Pulmonary Cryptococcosis" was published in 2022. Journal: Comput Math Methods Med.

# Clinical Diagnosis, Treatment, and Laboratory Detection of 50 Cases of Pulmonary Cryptococcosis

**DOI:** 10.1155/2022/7981472

**Published:** 2022-07-25

**Authors:** Tiantian Wang, Mulin Liu, Fenghua Zhang

**Affiliations:** ^1^Dalian Medical University, Dalian, 116044 Liaoning, China; ^2^Department of Laboratory Medicine, The First Affiliated Hospital of Dalian Medical University, Dalian, 116011 Liaoning, China; ^3^Department of Laboratory Medicine, Zhoupu Hospital Affiliated of Shanghai University of Medicine & Health Sciences, Shanghai 201318, China

## Abstract

**Objective:**

This study retrospectively analyzed the clinical diagnosis, treatment process, and laboratory test data of patients with pulmonary cryptococcosis to improve the understanding and diagnosis and treatment ability of the disease.

**Methods:**

Patients with pulmonary cryptococcosis diagnosed in the First Affiliated Hospital of Dalian Medical University from October 2003 to July 2021 were selected, and their medical records were consulted. The general data, clinical manifestations, laboratory examinations, imaging characteristics, diagnosis, and treatment methods were studied. The software SPSS 22 was used for statistical analysis.

**Results:**

A total of 50 patients with pulmonary cryptococcosis were included in the study. The ratio of male to female was 1 : 1. The average age was 53.56 ± 11.99 years with a range of 27-82 years. Grouping the patients by age, with 10 years as an age group, we found that 40-60 years was the high-incidence age group. Two patients (4%) had a history of bird contact, and 18 patients (36%) had at least one underlying conditions. Hypertension and cough were the most common underlying condition and clinical manifestation, respectively. The main admission diagnoses were lung shadow (19/50, 38%) and chest/lung mass (15/50, 30%). In the imaging findings, the most common type of lesions was nodule/nodule shadow (29/69, 42.03%). Lesion distribution in the lower lobe, single lobe, and right lung was more frequent than that in the upper lobe, multilobes, and left lung, respectively. Burr sign (12/43, 27.91%) was the most common concomitant sign. Pulmonary ventilatory defect was found in 7 cases. Laboratory test results were largely nonspecific. The pathological examination showed granuloma, with 47 cases (94%) confirmed by postoperative biopsy. Two cases (4%) were confirmed by serology. One case (2%) was diagnosed with *Cryptococcus* smear. 43 cases (86%) were treated with simple surgical resection, 6 cases (12%) were treated with antifungal drugs, and 1 case (2%) was transferred to another hospital for suspicion of pulmonary tuberculosis.

**Conclusions:**

Pulmonary cryptococcosis is more common in the middle-aged and elderly, and the clinical specificity is low. It can occur in people with normal or impaired immune function. The main clinical and imaging manifestation is cough and pulmonary nodules, which are very easy 5to be misdiagnosed. Surgical resection is the primary treatment.

## 1. Introduction

*Cryptococcus* is a genus of basidiomycetous fungi ubiquitously distributed in the environment. Although *Cryptococcus* has more than 30 species, only the *Cryptococcus neoformans* and *Cryptococcus gattii* are related to human diseases [1]. In China, cryptococcal infection is mainly caused by *Cryptococcus neoformans* [2]. This organism is typically found in soil and bird excreta, especially pigeon feces [3]. *Cryptococcus* can infect practically all organ systems, the most common of which are the central nervous system and the respiratory system with resultant cryptococcal meningitis and pulmonary cryptococcosis [4, 5]. The clinical manifestations of pulmonary cryptococcosis are subtle and nonspecific that renders early diagnosis difficult [6].

Pulmonary cryptococcosis is a type of respiratory mycosis caused by inhalation of *Cryptococcus* spores that can be acute, subacute, or chronic in disease presentation [7]. It has been considered that pulmonary cryptococcosis developed only in HIV-positive people with immune deficiency [8]. Nonetheless, studies reported increasing cases involving patients with normal immune function. According to a retrospective study in China, pulmonary cryptococcosis accounts for 60% of HIV-negative patients with normal immune function [9]. Patients with pulmonary cryptococcosis with different immune states have certain differences regarding clinical manifestations, laboratory test results, and imaging features [10–12]. *Cryptococcus* capsular antigen detection and pathological examination are the main methods for diagnosis, and surgical resection and antifungal medications are usually offered for treatment.

We retrospectively analyzed the clinical data of 50 patients with pulmonary cryptococcosis from the First Affiliated Hospital of Dalian Medical University. We aimed to sum up our experience and improve the understanding of pulmonary cryptococcosis by providing data from our department.

## 2. Materials and Methods

### 2.1. Study Subjects

Patients with pulmonary cryptococcosis admitted to the First Affiliated Hospital of Dalian Medical University from October 2003 to July 2021 were retrospectively selected. The study was approved by the Ethics Committee of the First Affiliated Hospital of Dalian Medical University (no. PJ-KS-KY-2021-276).

### 2.2. Data Collection

Patient data were retrieved from the electronic medical records. The following information was obtained: patient demographics, history of exposure to pigeons, underlying medical conditions, clinical manifestations, and imaging features on chest computed tomography. Blood test results, such as complete blood counts, erythrocyte sedimentation rate, C-reactive protein, tumor biomarkers carcinoembryonic antigen (CEA) and squamous cell carcinoma antigen (SCC), coagulation parameters, viral hepatitis biomarkers, treponema pallidum antibody, human immunodeficiency virus indicator, and biochemical parameters, were also recorded.

### 2.3. Diagnostic Method

A *Cryptococcus* capsular polysaccharide antigen was detected qualitatively, and ink staining was used for direct microscopic examination. The pathological methods of patients with pulmonary cryptococcosis, including thoracoscopic surgical resection, transbronchial lung biopsies, and percutaneous lung puncture, were recorded.

### 2.4. Pathological Features

The pathological characteristics of pulmonary cryptococcosis, including pathological type, special staining, and morphological characteristics, were observed under a light microscope.

### 2.5. Treatments

The treatment method, drug type, dose, administration route, and course of treatment were collected.

## 3. Results

### 3.1. Patient Demographics

Among the 50 patients included in the study, there were 25 males and 25 females with a male to female ratio of 1 : 1. The age range was 27-82 years, with an average age of 53.56 ± 11.99 years. The highest incidence was noted in patients with age between 40 and 60 years. The age distribution is shown in Table 1.

### 3.2. Susceptibility Factors

#### 3.2.1. Exposure History

Only 2 out of the 50 patients presented with a history of bird contact history.

#### 3.2.2. Underlying Medical Conditions

A total of 18 cases (36%) had at least one underlying medical condition, of which hypertension was the most common that was noted in 6 cases. The distribution of underlying medical conditions in these 18 patients is shown in Table 2.

### 3.3. Clinical Manifestations

#### 3.3.1. Types and Incidence of Clinical Manifestations

22 of the 50 patients had at least 1 of the following clinical manifestations, and the remaining 28 patients had no related clinical manifestations. The number of patients with cough, chest pain, chest tightness, shortness of breath, expectoration, blood in sputum, fever, fatigue, anorexia, pain around the body, dyspnea, and headache is shown in Table 3.

### 3.4. Preliminary Diagnosis

The 50 patients included in the statistics were not diagnosed accurately at the initial diagnosis. Preliminary diagnoses included lung shadow in 19 (38%), lung or chest mass in 15 (30%), pneumonia in 3 (6%), lung space-occupying lesions in 3 (6%), lung tumor in 2 (4%), pulmonary sarcoidosis in 1 (2%), undetermined shortness of breath in 1 (2%), and pulmonary tuberculosis in 1 (2%). The remaining 5 patients (10%) sought medical service for other diseases, and cryptococcosis was diagnosed at admission. The type and proportion of patients with corresponding preliminary diagnoses at admission are shown in Table 4.

### 3.5. Imaging Manifestations

#### 3.5.1. Lesion Shapes and Quantity

A total of 48 patients underwent imaging examinations, of which 69 lesions were observed, including nodule/nodule shadow in 29 cases, cord shadow/focus in 10 cases, miliary shadow/focus in 7 cases, pulmonary bullae in 5 cases, patch shadow in 4 cases, calcified focus in 3 cases, mass shadow in 3 cases, localized emphysema in 2, space-occupying lesions in 2, patch shadow in 2, mass shadow in 1, and leaf shadow in 1. The types and proportion of patients with varying imaging lesions are shown in Table 5.

#### 3.5.2. Lesion Distribution

Lesion distribution of the 48 patients with pulmonary cryptococcosis in the lower lobe, single lobe, and right lung was more than that in the upper lobe, multilobes, and left lung, respectively. The specific lesion location and distribution are shown in Table 6.

#### 3.5.3. Concomitant Signs

In imaging examination, 28 patients with pulmonary cryptococcosis showed one or more associated signs, including 12 cases of burr (27.91%), 7 cases of pleural thickening (16.28%), 5 cases of mediastinal lymph node enlargement (11.63%), 5 cases of lobulation (11.63%), 5 cases of cavity (11.63%), 3 cases of bronchitis sign (6.98%), 2 cases of pleural effusion (4.65%), 2 cases of vascular cluster sign (4.65%), 1 case of pleural depression sign (2.33%), and 1 case of spinous process (2.33%), as shown in Table 7.

### 3.6. Pulmonary Function Test

Among the 50 patients, 32 underwent pulmonary function tests, in which 25 (78.125%) were normal, 5 (15.625%) had obstructive ventilatory defect, and 2 (6.25%) had mixed ventilatory defect, as presented in Table 8.

### 3.7. Laboratory Test Results

#### 3.7.1. Blood Routine Test

The mean white blood cell count was 7.73 × 10^9^/L, in which 11 cases (22%) were high and 39 cases (78%) were normal. The mean lymphocyte count was 1.67 × 10^9^/L, in which 1 case (2%) was high, 44 cases (88%) were normal, and 5 cases (10%) were low. The mean neutrophil count was 5.39 × 10^9^/L, in which 15 cases (30%) were high and 35 cases (70%) were normal. The mean lymphocyte proportion was 25.25%, in which 2 cases (4%) were high, 31 cases (62%) were normal, and 17 cases (34%) were low. The mean proportion of neutrophils was 64.56%, in which 12 cases (24%) were high, 35 cases (70%) were normal, and 3 cases (6%) were low, as shown in Table 9.

#### 3.7.2. Inflammatory Indicators

Increased erythrocyte sedimentation rate was detected in 5 of the 29 cases measured (17.24%). Increased C-reactive protein was detected in 3 (25%) of the 12 cases measured, as shown in Table 10.

#### 3.7.3. Tumor Markers

The levels of CEA were measured in 45 of the 50 patients. Increased levels of CEA were found in only 2 cases (4.44%). Similarly, only 3 (11.11%) out of the 27 cases had elevated SCC, as shown in Table 11.

#### 3.7.4. Infectious Disease Inspection

Testing for hepatitis A antibody and hepatitis B surface antigen in 47 and 50 patients was all negative, respectively. In total, 9 cases (19.15%), 3 cases (6.38%), and 12 cases (25.53%) were positive for hepatitis B surface antibody, hepatitis B e antibody, and hepatitis B core antibody, respectively. All patients were negative for hepatitis C, and only 1 patient was positive for HIV (Table 12).

#### 3.7.5. Coagulation Indexes

Coagulation tests and D-dimer measurements were performed in 49 and 15 cases, respectively. Lower APTT, PT, and TT were noted in 4 (8.16%), 0 (0%), and 1 (2.04%), respectively. The mean value of FIB was 2.84 s, which was high in 4 cases (8.16%) and normal in 45 cases (91.84%). The mean value of D-dimer was 0.39 mg/L, which was high in 3 cases (20%) and normal in 12 cases (80%), as shown in Table 13.

#### 3.7.6. Biochemical Indexes

*(1) Blood Glucose*. Higher blood glucose and lower blood glucose were noted in 11 (22.92%) and 1 (2.08%) case out of the 48 cases tested, respectively (Table 14).

*(2) Blood Lipids*. As shown in Table 15, abnormal total cholesterol, triglyceride, high-density lipoprotein, and low-density lipoprotein were found in 6 (42.86%), 4 (28.57%), 5 (35.71%), and 4 (28.57%), respectively.

#### 3.7.7. Blood Group Detection

The ABO blood types tested in 35 patients were type A in 15 (42.86%), type B in 9 (25.71%), type AB in 2 (5.71%), and type O in 9 (25.71%). All the tested were Rh-positive (Table 16).

#### 3.7.8. Tuberculosis Antibody Test

Only 4 (18.18%) out of the 22 patients tested were weakly positive for tuberculosis antibody, as shown in Table 17.

### 3.8. Pathological Findings

Pathological examination predominantly showed granuloma that is histologically composed of multinucleated giant cells and epithelioid cells in a background of chronic fibrosis. Round fungi with transparent halo can be observed. In this study, 47 cases underwent pathological examination after invasive surgery. However, due to the age of the cases, the specific pathological manifestations of some patients were not recorded, and only 33 specific pathological manifestations were queried. The available 33 pathologic examinations were summarized, of which 22 cases (66.67%) reported directly cryptococcus, whereas granuloma and cryptococcus-like structures were reported in 6 (18.18%) and 5 cases (15.15%), respectively (Table 18).

### 3.9. Diagnostic Methods

As shown in Table 19, 47 cases were confirmed by pathological examination, including 43 cases of lobectomy, 1 case of pleural biopsy, 1 case of bronchial biopsy, and 2 cases of percutaneous lung biopsy. The other 3 cases were diagnosed by cryptococcus capsular antigen in 2 cases and cryptococcus smear in 1 case.

### 3.10. Treatment Plan

A total of 43 cases and 6 cases were treated by surgical resection and antifungal medications that are predominantly composed of fluconazole, respectively (Table 20). The other case was transferred to another hospital for high suspicion of concomitant pulmonary tuberculosis.

## 4. Discussion

Cryptococci causing human infections are mainly *Cryptococcus neoformans* and *Cryptococcus gattii* [13]. Cryptococcal infection can occur in multiple organs, particularly the central nervous system, the lungs, the skin, and the bones, in a decreasing order of frequency. *Cryptococcus* is widely distributed and can appear in pigeon dung, soil, vegetables, fruits, and air [11]. Close contact with pigeons or pigeon dung is a factor for cryptococcosis. Similar to a previous report, only 2 cases (4%) have a documented history of pigeon contact in this study [14], suggesting that environmental exposure may not be the main cause of pulmonary cryptococcosis. However, the physician should be highly vigilant for pulmonary cryptococcosis in a patient with history of pigeon contact accompanied by clinical symptoms and expectoration.

Similar to the literature [6], most of the underlying diseases were malignant tumors and diabetes, which may be related to their detrimental effect to the integrity of human immunity. At the same time, the literature [15] has shown that diabetes has become an independent factor for mortality in patients with cryptococcosis.

According to immune status, we divided patients into immunocompetent and immunocompromised groups [12, 16, 17]. In the immunocompetent group, no recognized underlying disease exists or the underlying disease does not affect immunity, such as hypertension. The immunocompromised group must meet one of the following medical histories: long-term use of immunosuppressive drugs or glucocorticoid therapy, diabetes, malignancy, HIV infection, decompensated liver cirrhosis, organ transplantation, acquired immunodeficiency syndrome, idiopathic CD4 lymphocytosis, agranulocytosis, and other conditions that cause severe immunosuppression or other systemic diseases (e.g., systemic lupus erythematosus). In this study, we found that 12 (24%) patients with pulmonary cryptococcosis were immunocompromised, and 38 (76%) pulmonary cryptococcosis patients with normal immunity had results similar to those reported in the literature [16]. It shows that pulmonary cryptococcosis can also occur in people with normal immunity, and the incidence is increased in people with normal immunity [10].

In this study, 28 patients had no clinical manifestations, and 22 patients had one or more of the following clinical manifestations: cough, chest pain, chest tightness, shortness of breath, expectoration, blood in sputum, fever, fatigue, anorexia, body pain, dyspnea, and headache. This study found that the clinical manifestations in 22 patients were nonspecific and difficult to be differentiated from tumors, inflammations, and other lesions. It can be concluded that the clinical manifestations of pulmonary cryptococcosis are heterogeneous and nonspecific [10, 18].

The results of this study showed that the lesions of pulmonary cryptococcosis involved the right lung and the lower lobe more frequently than the left lung and the middle and upper lobe, respectively. Single or multiple nodules accounting for 42.03% were the most common imaging findings. The results were consistent with those reported in the literature [10, 18, 19]. The literature [16] showed certain differences in imaging manifestations in patients with different immune status. The chest CT manifestations of patients without clinical symptoms were mostly of localized nodule/mass type, while those in immunosuppressive patients were pneumonia type and mixed type. However, no differences in imaging manifestations of patients with different immune status were found in this study, which is the same as reported in previous reports [20]. This disparity may be related to small sample size, geographic differences, and the extent of immunity compromise. In this study, the pulmonary lesions of 48 patients were of different shapes, and no characteristic lesions were found, rendering clinical diagnosis and treatment difficult. Therefore, imaging manifestations have a certain significance for the diagnosis of pulmonary cryptococcosis and should be interpreted with an appropriate clinical scenario. However, it should also be noted that imaging manifestations of pulmonary cryptococcosis needs to be differentiated from peripheral lung cancer, pulmonary metastatic cancer, and pulmonary tuberculosis [18].

In addition to the above imaging findings, pulmonary cryptococcosis also showed burr, pleural thickening, mediastinal lymph node enlargement, lobulation sign, cavity, bronchitis sign, pleural effusion, vascular convergence sign, pleural depression sign, and spinous process, with burr the most common in this study. In addition, it was found that nodular type was mostly accompanied by burr and lobulation. However, this imaging manifestation is similar to that of lung cancer, making differential diagnosis and treatment difficult [18]. Fewer pleural effusions were found in this study, with only 2 cases. The reason may be that the inflammatory granulomatous lesions of the fungus itself do not lead to large-scale inflammation and necrosis, and it is difficult to lead to the production of exudative pleural effusion.

This study showed that the laboratory examination of pulmonary cryptococcosis had no specificity, which is compatible with an earlier report [13]. This study showed that the leukocyte and neutrophil count was increased, which may be explained by the fact that neutrophils have certain phagocytosis and toxic effects on *Cryptococcus* [21]. In our study, erythrocyte sedimentation rate and C-reactive protein were increased in 5 cases (17.24%) and 3 cases (25%), respectively, which may be caused by cryptococcal infection. In this study, it was also observed that the blood lipid of some patients increased slightly, a phenomenon probably related to the advanced age and coexistence of hypertension in this cohort. The blood routine, erythrocyte sedimentation rate, tumor markers, coagulation indexes, biochemical indexes, and other related indexes in most patients were within the normal range. This suggested that cryptococcal infection does not produce an acute response, which can be differentiated from bacterial pneumonia. This study showed that most patients (88.89%) had SCC in the normal range. Literature [22] suggests that the level of SCC in patients with lung cancer is higher than that in patients with benign lung diseases and healthy people, indicating its potential utility for the ancillary diagnosis of lung cancer. The finding that some patients tested positive for the tuberculosis antibody may also be related to a previous infection.

Although 47 patients were diagnosed with pulmonary cryptococcosis by pathological examination, due to the large time span of patient cases, the detailed pathological manifestations of some patients were not recorded, and only the specific pathological manifestations of 33 patients were queried. Among them, 22 cases (66.67%) described seeing *Cryptococcus*. Granuloma (*Cryptococcus*) was described in 6 cases (18.18%). *Cryptococcus*-like structures in multinucleated giant cells were described in 5 cases (15.15%).

Concerning the diagnosis of pulmonary cryptococcosis in this cohort, 47 patients (94%) were diagnosed by “gold standard” pathology [17]. Granulomatous inflammation with light blue or colorless bacteria that were positive for PAS staining suggested cryptococcal infection. Among them, 43 cases underwent lobectomy, 1 case underwent pleural biopsy, 1 case underwent bronchial biopsy, 2 cases underwent percutaneous lung biopsy, 2 cases were confirmed by serology, and a cryptococcal capsular antigen was positive with pulmonary lesions. One case was diagnosed with *Cryptococcus* smear.

Among them, percutaneous lung biopsy is performed under X-ray fluoroscopy, ultrasound, or CT that uses a fine needle to extract lesion tissue for pathological examination. This method is safe, fast, and accurate with a high positive rate and minimal trauma. However, only 4% of the patients were diagnosed by percutaneous lung biopsy in this study. The main reason is that most of the patients were suspected of malignant lung tumors before the operation and underwent surgical resection.

Ink staining is one of the most commonly used methods for the diagnosis of *Cryptococcus*. However, the positive rate is low and limited by mixed cells and fat droplets. Moreover, the sensitivity of ink staining in the early stage is also not high. Thus, it needs to be detected together with other detection methods, which can improve the diagnostic rate. The diagnosis of pulmonary cryptococcosis by ink staining is simple and rapid. Still, its detection sensitivity is easily affected by many factors, such as the number of fungus in the sample, the treatment method (centrifugation speed and time), the experience of the tester, and whether the subject is HIV infected.

Detection of the *Cryptococcus* capsular polysaccharide antigen is carried out using a colloidal gold method. It has the characteristics of low cost, easy operation, fast detection time, and high sensitivity and specificity. The detection of the cryptococcal capsular polysaccharide antigen has high diagnostic and differential diagnostic value in diagnosing and treating pulmonary cryptococcosis [23, 24]. Compared with surgical resection, detecting the *Cryptococcus* capsular polysaccharide antigen has the advantages of simplicity, rapidity, and low damage. The detection of the *Cryptococcus* capsular polysaccharide antigen should be advocated in patients suspected of pulmonary *Cryptococcus* to avoid traumatic biopsy.

In the present study, pulmonary cryptococcosis was not diagnosed initially, and most of the patients were eventually proven to be misdiagnosed as reported previously [23, 25]. Pulmonary cryptococcosis is challenging to diagnose due to the lack of specific clinical symptoms and generally insufficient experience. Some patients were misdiagnosed with lung cancer and underwent surgical resection that caused unnecessary damage. Therefore, it is particularly important to improve the experience and awareness of pulmonary cryptococcosis.

The goal of pulmonary cryptococcosis treatment is to control and prevent the spread of infection. The treatment scheme is determined by the immune status and disease severity. The expert consensus for the diagnosis and treatment of cryptococcal infection recommended that patients with normal immunity and asymptomatic patients must be closely observed or treated with fluconazole, 200~400 mg per day for 3~6 months. Patients with normal immunity and mild to moderate symptoms or those with nonsevere immunosuppression and diffuse lung infiltration or those with involvement of other systems should be treated with fluconazole, 200~400 mg per day for 6~12 months. For patients who cannot tolerate fluconazole, itraconazole, 200~400 mg per day, can be used for 6~12 months. For those who underwent surgical resection due to thoracotomy exploration or misdiagnosis as tumors or other lesions, it is recommended to apply antifungal drugs routinely after the operation. The course of treatment should not be less than 2 months. Most patients in this study, 43 (86%), underwent surgical resection due to thoracotomy or were misdiagnosed with lung cancer or other lesions. The prognosis of all patients after operation was good, the condition was stable, and the clinical symptoms were greatly relieved, mainly because the lesions were simply limited. When antifungal drugs were used for an average of about 13 days, the clinical symptoms of most patients were significantly relieved. According to the results of this study, the main treatment methods for pulmonary cryptococcosis are surgical resection and antifungal drug treatment. The prognosis is favorable with remarkable treatment effect.

## Figures and Tables

**Table 1:** Age distribution of patients with pulmonary cryptococcosis.

Group	Male	Female	Total
20-29	1 (2%)	0 (0%)	1 (2%)
30-39	2 (4%)	1 (2%)	3 (6%)
40-49	7 (14%)	8 (16%)	15 (30%)
50-59	7 (14%)	9 (18%)	16 (32%)
60-69	4 (8%)	6 (12%)	10 (20%)
70-79	2 (4%)	1 (2%)	3 (6%)
80-89	2 (4%)	0 (0%)	2 (4%)
Total	25 (50%)	25 (50%)	50 (100%)

**Table 2:** Distribution of basic diseases in 18 patients with pulmonary cryptococcosis.

	Underlying medical conditions
Case 1	Hypothyroidism, thyroiditis, metabolic disorder, uremia
Case 2	Hypertension (grade I), coronary heart disease
Case 3	Hypertension (grade II), fatty liver, hyperlipidemia
Case 4	Type 2 diabetes
Case 5	Type 2 diabetes
Case 6	Hypertension (grade II), low incomplete intestinal obstruction
Case 7	Cryptococcal meningitis
Case 8	Diabetes (grade II)
Case 9	Hypertension, diabetes
Case 10	Lung cancer
Case 11	Benign prostate hyperplasia, polycythemia, bone marrow proliferative tumor
Case 12	Serpentine ulcer, lung cancer
Case 13	Pneumonia, tuberculosis
Case 14	Malignant tumor
Case 15	Malignant tumor of lung
Case 16	Hypertension (grade III), rheumatoid arthritis, renal insufficiency, atherosclerosis
Case 17	Type 2 diabetes
Case 18	Hypertension (grade II), hypoxic hypercapnia, asthma, COPD overlap syndrome, malignant tumor

**Table 3:** Types and incidence of clinical manifestations.

Clinical manifestations	Number of cases	Incidence (%)
Cough	13	26
Chest pain	8	16
Chest tightness	8	16
Shortness of breath	5	10
Expectoration	5	10
Bloody sputum	2	4
Fever	2	4
Weakness	2	4
Poor appetite	1	2
Generalized aches and pains	1	2
Dyspnea	1	2
Headache	1	2

**Table 4:** Types and proportion of preliminary diagnosis.

Type	Case	Proportion (%)
Lung shadow	19	38
Lung or chest mass	15	30
Pneumonia	3	6
Lung space-occupying lesion	3	6
Lung tumor	2	4
Pulmonary sarcoidosis	1	2
Shortness of breath	1	2
Pulmonary tuberculosis	1	2
Other	5	10
Total	50	100

**Table 5:** Types and proportion of patients with pulmonary cryptococcus.

Lesion type	Case	Proportion (%)
Nodule/nodule shadow	29	42.03
Cord shadow/focus	10	14.49
Miliary shadow/focus	7	10.14
Pulmonary bullae	5	7.25
Patch shadow	4	5.80
Calcified focus	3	4.35
Mass shadow	3	4.35
Localized emphysema	2	2.90
Seize a seat	2	2.90
Flake shadow	2	2.90
Mass shadow	1	1.45
Leaf shadow	1	1.45
Total	69	100

**Table 6:** Distribution of lesions in patients with pulmonary cryptococcus.

Position	Left lung	Right lung	Both lungs	Total
Upper lobe	2	4	2	8
Middle lobe		1		1
Lower lobe	4	9	4	17
Multilobes	0	6	16	22
Total	6	20	22	48

**Table 7:** Imaging concomitant signs in patients with pulmonary cryptococcosis.

Concomitant sign	Case	Proportion (%)
Burrs	12	27.91
Pleural thickening	7	16.28
Mediastinal lymph node enlargement	5	11.63
Lobulation	5	11.63
Cavity	5	11.63
Bronchitis	3	6.98
Pleural effusion	2	4.65
Vascular cluster sign	2	4.65
Pleural depression sign	1	2.33
Spinous process	1	2.33
Total	43	100

**Table 8:** Pulmonary ventilation function.

Pulmonary ventilation function	Case	Proportion (%)
Normal pulmonary ventilation function	25	78.125
Obstructive pulmonary ventilation dysfunction	5	15.625

Mixed pulmonary ventilation dysfunction	2	6.25

**Table 9:** Blood routine examination.

Blood test	Normal value	Average	Higher	Normal	Lower
Leukocyte count	3.5-9.5 (10^9^/L)	7.73 (10^9^/L)	11 (22%)	39 (78%)	0 (0%)
Lymphocyte count	1.1-3.2 (10^9^/L)	1.67 (10^9^/L)	1 (2%)	44 (88%)	5 (10%)
Neutrophil count	1.8-6.3 (10^9^/L)	5.39 (10^9^/L)	15 (30%)	35 (70%)	0 (0%)
Lymphocyte ratio	20-50 (%)	25.25 (%)	2 (4%)	31 (62%)	17 (34%)
Proportion of neutrophils	45-75 (%)	64.56 (%)	12 (24%)	35 (70%)	3 (6%)

**Table 10:** Examination results of inflammatory indexes.

Inflammatory indicators	Normal value	Higher	Normal
Erythrocyte sedimentation	0-20 (mm/h)	5 cases (17.24%)	24 cases (82.76%)
CRP	0-8 (mg/L)	3 cases (25%)	9 cases (75%)

**Table 11:** Examination results of tumor markers.

Tumor markers	Normal value	Average	Higher	Normal
CEA	0-5 (ng/mL)	1.89	2 cases (4.44%)	43 cases (95.56%)
SCC	0-2.5 (ng/mL)	1.28	3 cases (11.11%)	24 cases (88.89%)

**Table 12:** Inspection results of infectious diseases.

Infectious disease indicators	Negative	Positive	Total
Anti-HAV antibody	47 (100%)	0 (0%)	47 (100%)
HBsAg	50 (100%)	0 (0%)	50 (100%)
Anti-HBsAg antibody	38 (80.85%)	9 (19.15%)	47 (100%)
HBeAg	47 (100%)	0 (0%)	47 (100%)
Anti-HbeAg antibody	44 (93.61%)	3 (6.38%)	47 (100%)
Anti-HbcAg antibody	35 (74.47%)	12 (25.53%)	47 (100%)
PreS1	47 (100%)	0 (0%)	47 (100%)
Anti-HCV antibody	50 (100%)	0 (0%)	50 (100%)
Anti-HEV antibody	47 (100%)	0 (0%)	47 (100%)
Anti-TP antibody	50 (100%)	0 (0%)	50 (100%)
HIV	47 (97.92%)	1 (2.08%)	48 (100%)

**Table 13:** Examination results of coagulation indexes.

Coagulation indexes	Normal value	Average	Higher	Normal	Lower
APTT	19-31 (s)	23.58	0 (0%)	45 (91.83%)	4 (8.16%)
PT	9-13 (s)	10.77	0 (0%)	49 (100%)	0 (0%)
TT	14-20 (s)	16.80	0 (0%)	48 (97.96%)	1 (2.04%)
Fib	1.8-3.9 (g/L)	2.84	4 (8.16%)	45 (91.84%)	0 (0%)
D-dimer	<0.55 (mg/L FEU)	0.39	3 (20%)	12 (80%)	0 (0%)

**Table 14:** Glucose test results.

Biochemical indexes	Normal value	Average	Higher	Normal	Lower
Glucose	3.9-6.1 (mmol)	5.915	11 cases (22.92%)	36 cases (75%)	1 case (2.08%)

**Table 15:** Blood lipid test results.

Blood lipids	Normal value	Normal	Abnormal
TC	<5.20 (mmol/L)	8 (57.14%)	6 (42.86%)
TG	<1.70 (mmol/L)	10 (71.43%)	4 (28.57%)
HDL	>1.04 (mmol/L)	9 (64.28%)	5 (35.71%)
LDL	<3.12 (mmol/L)	10 (71.43%)	4 (28.57%)

**Table 16:** Blood group test results.

Blood types	Cases	Proportion (%)
A	15	42.86
B	9	25.71
AB	2	5.71
O	9	25.71
Rh (+)	35	100

**Table 17:** TB antibody test results and proportion.

Test results	Cases	Proportion (%)
Negative	18	81.82
Weakly positive	4	18.18

**Table 18:** Pathological manifestations of pulmonary cryptococcosis.

Pathological findings	Cases	Proportion (%)
*Cryptococcus* was found	22	66.67
Granuloma	6	18.18
*Cryptococcus*-like structure in multinucleated giant cells	5	15.15

**Table 19:** Diagnostic methods.

Diagnostic methods	Cases	Proportion (%)
Pathological examination	47	94
Cryptococcus capsular antigen	2	4
Cryptococcus smear	1	2

**Table 20:** Treatment plan.

Treatment plan	Cases
Resection	43
Antifungal drugs	6

## Data Availability

The data used to support the findings of this study are included within the article.
